The article "Application of ICH Guidelines for the Assessment and Control of Elemental Impurities in Parecoxib Sodium by Graphite-Digestion and ICP-MS" was published in 2022. Journal: Int J Anal Chem.

# Application of ICH Guidelines for the Assessment and Control of Elemental Impurities in Parecoxib Sodium by Graphite-Digestion and ICP-MS

**DOI:** 10.1155/2022/9299416

**Published:** 2022-08-24

**Authors:** Yajie Hao, Guang Yin, Xuemei Wang, Zhenglei Jiang, Guimin Zhang, Zhong Feng, Qinyong Sun

**Affiliations:** ^1^Department of International Pharmaceutical R&D Centre, Lunan Pharmaceutical Group, 1 North Outer Ring Road, Fei County, Linyi City, Shandong, China; ^2^School of Pharmaceutical Sciences (Shenzhen), Sun Yat-Sen University, Shenzhen, China

## Abstract

Parecoxib sodium is a widely used parenteral cyclooxygenase 2 selective inhibitor to relieve acute postoperative pain following gynecologic laparotomy surgery. To ensure the quality of the drug, a detailed quality specification is indispensable. Nevertheless, it is unavoidable to introduce inorganic impurities during the drug preparation process and how to assess and control them matters. This study proposed an analytical procedure for the determination of elemental impurities (Cd, Pb, As, Hg, Co, V, Ni, Li, Sb, and Cu) in parecoxib sodium, where an easier and safer digestion protocol, graphite digestion, combined with an inductively coupled plasma-mass spectrometer (ICP-MS) was adopted when compared with microwave digestion. Moreover, the study also discussed whether should they be listed in specification to comply with ICH Q3D guidelines after test of process validation batches. Limit of quantitation (LOQ) of the above elemental impurities reached to 0.05, 0.125, 0.375, 0.075, 0.125, 0.25, 0.5, 6.25, 2.25 and 7.5 ppm, respectively, and recovery in accuracy item ranged from 90.2% to 129.9%, reflecting a sensitive and accurate method.

## 1. Introduction

Parecoxib sodium, which served as an injectable COX-2-specific inhibitor, was extensively employed for the analgesic efficacy and safety of single intravenous doses to relieve acute postoperative pain in patients after gynecologic laparotomy surgery [1–3]. Given the presence of impurities, even in small amounts, which may affect drug safety and efficacy [4], much more importance should be attached to the quality control of parecoxib sodium, especially impurities control in raw material. Impurities can be classified into organic impurities (process-and drug-related), inorganic impurities as well as residual solvents, and all of those can result from the manufacturing process [4–6]. Take inorganic impurities, for example, they root in reagents, ligands, catalysts, heavy metals or other residual metals, inorganic salts, and other materials that are used in the formation of parecoxib sodium and do not provide any therapeutic benefit to the patient. Therefore, the control of elemental impurities introduced through the preparation of parecoxib sodium is of great significance in ensuring the quality of the product.

Analysis of elemental impurities in drugs, foods, plants, and crude oil using microwave oven digestion combined with an inductively coupled plasma-mass spectrometer (ICP-MS) has been previously reported though [7–11], there are limited reports about elemental impurities in drugs analyzed by a none microwave oven digestion combined with ICP-MS due to the complex structures of analytes, like parecoxib sodium, in the form of salt (Figure 1). Microwave oven digestion is an effective way but it is time-consuming and not safe. On one hand, it will take at least 2 hours to digest samples. On the other hand, the high pressure is up to 100–150 bar and the temperature is up to 180–240°C in the process of microwave digestion. Our team proposed graphite digestion, a 30 minutes process, coupled with the ICP-MS method to measure elemental impurities in parecoxib sodium.

Based on the manufacturing process of parecoxib sodium and ICH Q3D guidelines, 10 selected elemental impurities, including Cd, Pb, As, Hg, Co, V, Ni, Li, Sb, and Cu, should be considered and controlled within acceptable limits after a risk assessment [12, 13]. The limit concentration of above 10 elements were 0.2, 0.5, 1.5, 0.3, 0.5, 1, 2, 25, 9, and 30 ppm. The analytical procedure was developed and validated.

## 2. Materials and Methods

### 2.1. Materials and Standards

Deionized water produced by a Milli-Q Integral 10 system (Merck, Germany) was used to prepare all solutions. Optima grade concentrated nitric acid (Fisher scientific chemical, USA) and analytical reagent 30% (m/m) hydrogen peroxide (Xilong Scientific, China) were employed in the sample preparation. ICP Multi-Element standard (5 elements, Bi, In, Sc, Tb, and Y at 100 mg/L in 2% (v/v) HNO_3_) was purchased from Reagecon (Ireland). ICP standard cadmium 1000 mg/L, ICP standard Lead 1000 mg/L, ICP standard arsenic 1000 mg/L, ICP standard cobalt 1000 mg/L, ICP standard vanadium 1000 mg/L, ICP standard nickel 1000 mg/L, ICP standard copper 1000 mg/L, and ICP standard lithium 1000 mg/L were purchased from Reagecon (Ireland). ICP standard mercury 1000 mg/L, ICP standard antimony 1000 mg/L, and ICP standard gold 1000 mg/L were obtained from National Non-ferrous Metals and Electronic Materials Analysis Center (China). Argon (99.999%) and helium (99.999%) gases were provided by Jinan Deyang Special Gas Co., LTD. (Shangdong, China). Parecoxib sodium was obtained from New Time Pharmaceutical Co. Ltd, Shang Dong, China.

### 2.2. Standard Solutions

Internal standard solution at a concentration of 25 *μ*g/L was prepared by serial dilutions of ICP Multi-Element standard in 10% (v/v) HNO_3_. The standard stock solution was prepared by dilutions of 10 ICP standard elements into a mixture in 10% (v/v) HNO_3_, containing 0.04 mg/L of Cd, 0.1 mg/L of Pb, 0.3 mg/L of As, 0.06 mg/L of Hg, 0.1 mg/L of Co, 0.2 mg/L of V, 0.4 mg/L of Ni, 5 mg/L of Li, 1.8 mg/L of Sb, and 6 mg/L of Cu. The standard solution was prepared by diluting 0.25 mL standard stock solution plus 20 *μ*L ICP standard Gold 1000 mg/L into 25 mL in 10% (v/v) HNO_3_. All plastic volumetric apparatus used were immersed in 10% (v/v) HNO_3_ for 24 h and rinsed with deionized water.

### 2.3. Preparation of the Sample and Spiked Sample by Graphite Digestion

#### 2.3.1. Sample

Parecoxib sodium (0.05 g, 0.127 mmol) was weighted accurately and placed in a digestion tank; 3 mL of nitric acid, 20 *μ*L of ICP standard gold 1000 mg/L, and 3 mL of 30% (m/m) hydrogen peroxide were then added into the tank. After mixed, they were heated on a graphite furnace (Laboratory, China) at 100°C for 30 min and transferred into a 25 mL plastic volumetric flask after cooling. Finally, they were diluted with deionized water to volume and mixed.

#### 2.3.2. Spiked Sample

Parecoxib sodium (0.05 g, 0.127 mmol) was weighted accurately and placed in a digestion tank; 3 mL of nitric acid, 20 *μ*L of ICP standard gold 1000 mg/L, 3 mL of 30% (m/m) hydrogen peroxide, and 0.25 mL of standard stock solution were then added into the tank. After mixed, they were heated on a graphite furnace at 100°C for 30 min and transferred into a 25 mL plastic volumetric flask after cooling. Finally, they were diluted with deionized water to volume and mixed.

### 2.4. Inductively Coupled Plasma-Mass Spectrometry Conditions

ICP-MS experiments were carried out using an iCAP RQ mass spectrometer (Thermo Fisher Scientific, USA) equipped with an ASX-560 autosampler (Teledyne Cetac Technologies). Argon was used for plasma generation and worked as nebulization and auxiliary gas. Helium was used as collision gas. Plasma power was set as 1550 W, uptake time 80 seconds at a rate of 40 rpm/min, wash time 60 seconds, a number of sweeps 20 times, main runs 3 times, plasma gas 14 L/min, Nebulizer gas 5.4 mL/min, and Auxiliary gas 0.8 L/min. The most abundant isotopes, 111Cd+, 208 Pb+, 75 As^+^, 202Hg^+^, 59Co^+^, 51V^+^, 60Ni^+^, 7Li^+^, 121Sb^+^, and 65Cu^+^, were determined in kinetic energy discrimination (KED) mode. 209Bi^+^, 115In^+^, 45Sc^+^ and 89Y^+^ were determined in KED mode as internal standards. Dwell time was 0.1 seconds and resolution were selected as normal.

### 2.5. Method Validation and Sample Test

The method was validated as a quantitative procedure to determine elemental impurities in parecoxib sodium and system suitability, specificity, linearity, the limit of quantitation, solutions stability, accuracy as well as precision of the method were monitored. System suitability was determined using the injection of standard solution, every 9 injections, to evaluate the relative standard deviation (RSD%). Specificity was determined by injecting blank, standard solution, sample, and spiked sample solutions to observe the interference of diluent and sample. Linearity was performed by preparing standard solutions of different concentration levels (levels 1–5), including 25%, 50%, 100%, 150%, and 250% standard solutions, and determined by constructing the calibration plots by taking standard solutions of above concentration levels. The stability of both spiked sample and the standard solution was tested for 4 h using freshly prepared solutions at room temperature. For the investigation of stability, each solution was injected into the ICP-MS system and analyzed for intact elements. Changing rate of these samples was compared to that of freshly prepared samples to determine solutions stability. Accuracy was assessed by the recoveries of spiking solutions with drugs corresponding to three concentration levels (50, 100, and 150%), recorded for each concentration in triplicate. Precision was demonstrated by interday and intraday studies on spiked sample solutions in sextuplicate, via calculating the standard deviations and %RSD of recoveries.

## 3. Results and Discussion

### 3.1. Optimization of Graphite Digestion

The final digestion condition was selected after several experiments with different digestion processes. Initially, 5 mL of nitric acid plus 2 mL of 30% (m/m) hydrogen peroxide were added to 0.1 g parecoxib sodium, the liquid mixture stayed clear after being heated in a graphite furnace at 100°C for 30 min. Nevertheless, it cost a lot of nitric acid and a higher concentration of nitric acid did harm to the environment, minor nitric acid was preferable. When the volume of nitric acid was reduced to 2 mL and other parameters remained, the liquid mixture went from clear to muddy left overnight. Then, 2 mL of nitric acid plus 2 mL of 30% (m/m) hydrogen peroxide were added to 0.05 g parecoxib sodium, the liquid mixture was clear after being heated in a graphite furnace at 100°C for 30 min and went from clear to muddy left overnight, which indicated that 2 mL of nitric acid was not sufficient to digest 0.05 g parecoxib sodium. Finally, 3 mL of nitric acid plus 3 mL of 30% (m/m) hydrogen peroxide were added into 0.05 g parecoxib sodium, the liquid mixture stayed clear after heated on graphite furnace at 100°C for 30 min. To prevent recovery of Hg from being lower than 70% caused by volatilization in digestion, 20 *μ*L of ICP standard gold 1000 mg/L was added before heating, ultimately.

### 3.2. Determination of Standard Solution Concentration

By ICH Q3D guidelines, parenteral permitted daily exposures for elemental impurities (Cd, Pb, As, Hg, Co, V, Ni, Li, Sb, and Cu) should be 2, 5, 15, 3, 5, 10, 20, 250, 90, and 300 micrograms per day (Table 1). Moreover, option 1 was selected to assess the elemental impurity content in drug substances with daily doses of not more than 10 grams per day [12]. Consequently, the values represent permitted concentrations in micrograms per gram for above elemental impurities were 0.2, 0.5, 1.5, 0.3, 0.5, 1, 2, 25, 9, and 30 *μ*g/g, respectively. When the concentration of the parecoxib sodium sample was confirmed (2 mg/mL), the standard solution concentration could be calculated. Furthermore, sample, spiked sample, and standard solution were injected into ICP-MS to evaluate the sensitivity and accuracy of the method preliminarily. Once responses of the elemental impurities to be measured were too low to test, a higher concentration of standard solution would be necessary. Moreover, if recoveries of the elemental impurities calculated were out of the specified range (70%–150%), further optimization of graphite digestion should be carried out.

### 3.3. Method Validation

The developed method was validated as per ICH guidelines for analytical performance parameters including system suitability, specificity, linearity, the limit of quantitation, accuracy, precision, and solutions stability. Moreover, the results showed a selective, highly sensitive, accurate, and reproducible method.

#### 3.3.1. System Suitability

System suitability parameters were evaluated from standard solutions every 9 injections in sample list. The % RSD of 10 elements (Cd, Pb, As, Hg, Co, V, Ni, Li, Sb, and Cu) intensities from five replicated injections were 1.4%, 4.4%, 3.2%, 3.6%, 3.3%, 4.2%, 3.8%, 3.9%, 4.0% and 2.7%, respectively, and satisfy the system suitability parameters (%RSD of intensities NMT 20%), which showed a stable system and that validation could be continued.

#### 3.3.2. Specificity

The specificity of the method was determined from blank, sample, and spiked sample, and standard solutions revealed that there were no other impurities intensity or interference found in each individual analyte selected; hence, it implied the developed method was a specific method.

#### 3.3.3. Linearity

The method linearity was determined from regression equations *f* (*x*) = 142.8612 *x* + 2.8318 for Li, *f* (*x*) = 13957.8354 *x* + 39.3971 for V, *f* (*x*) = 41037.1883 *x* + 51.79 for Co, *f* (*x*) = 11106.8984 *x* + 1350.5993 for Ni, *f* (*x*) = 27747.0868 *x* + 1395.775 for Cu, *f* (*x*) = 1288.2543 *x* + 8.1465 for As, *f* (*x*) = 5711.2262 *x* + 9.5109 for Cd, *f* (*x*) = 9127.4006 *x* + 41.9995 for Sb, *f* (*x*) = 14472.4198 *x* + 209.8530 for Hg, and *f* (*x*) = 102465.0097 *x* + 2135.6275 for Pb (f (*x*) = *ax* + *b*), obtained from calibration curves. The obtained calibration plots are depicted in Figure 2. The correlation coefficient was found to be 0.9999 for Li, 0.9999 for V, 0.9998 for Co, 0.9994 for Ni, 0.9999 for Cu, 0.9999 for As, 0.9999 for Cd, 0.9999 for Sb, 0.9998 for Hg and 0.9980 for Pb, greater than 0.99, which indicated good linearity.

#### 3.3.4. Limit of Quantitation

It was observed that LOQ values for elements Cd, Pb, As, Hg, Co, V, Ni, Li, Sb, and Cu in this method were 0.1, 0.25, 0.75, 0.15, 0.25, 0.5, 1, 12.5, 4.5 and 15 *μ*g/L, respectively. The procedure described that the framework for the quantification of the 10 elements had a reasonably high sensitivity.

#### 3.3.5. Accuracy

The accuracy studies were performed for three concentration levels: 50, 100, and 150%. The mean percentage recovery of Cd was 92.8%, Pb was 104.0%, As was 115.6%, Hg was 105.7%, Co was 104.3%, V was 111.1%, Ni was 107.3%, Li was 110.0%, Sb was 94.1%, Cu was 103.1%, and all found to be within the permissible limits ranged from 70% to 150%, which showed that the proposed method was accurate. The data of recovery studies are presented in Table 2.

#### 3.3.6. Precision

The precision of the analytical method was demonstrated by interday and intraday studies (repeatability and reproducibility) by calculating the recoveries of 10 elements in each injection as well as their % RSD. % RSD of recoveries was found to be 2.0 (Cd), 1.8 (Pb), 1.6 (As), 2.0 (Hg), 1.7 (Co), 1.7 (V), 2.2 (Ni), 1.2 (Li), 1.2 (Sb), and 2.1 (Cu). The value of % RSD in all samples were less than 20, and the results are presented in Table 3.

#### 3.3.7. Stability

The stability of both spiked sample and standard solution were tested over a period of 4 h using freshly prepared solutions at room temperature. For the investigation of stability, each solution was injected into the ICP-MS system and analyzed for intact compounds. Intensities changing rate of these elements compared to that of freshly prepared samples ranged from 0.2% to 9.3%, not more than 20%, which manifested solutions were stable.

### 3.4. Sample Testing

The validated procedure was adopted to detect elemental impurities in 3 process validation batches and 3 commercial batches. Impurities of all batches were less than 30% of permitted daily exposure that was defined as the control threshold, indicating additional controls were not required in the specification by ICH Q3D and ICH Q6 guidelines for the data had been assessed appropriately and controls on elemental impurities demonstrated adequately [12, 14]. If the risk assessment failed to demonstrate that an elemental impurity level was consistently less than the control threshold, controls should be established to ensure that the elemental impurity level did not exceed the PDE in the drug.

## 4. Conclusions

The linearity, specificity, precision, and recovery found according to ICH guidelines and the development of a graphite-digestion combined with an ICP-MS system for quantitative elemental impurities measurement in parecoxib sodium have been validated. In addition, this article has expanded on how to evaluate the elemental impurities and determine the limit on the base of ICH Q3D and whether the control of elemental impurities should be defined in drug specification.

Moreover, the procedure was easier with regard to a briefer operation and shorter duration and safer without a higher pressure compared with microwave digestion, allowing this analytical approach for elemental impurities quantification in drug substances to be used efficiently and conveniently.

## Figures and Tables

**Figure 1:** Structure of parecoxib sodium.

**Figure 2:** Linearity calibration plots of elements Li, V Co, Cu, As, Cd, Sb, Hg, and Pb.

**Table 1:** Permitted daily exposures for elemental impurities established in ICH Q3D.

Element	Class	Oral PDE,*μ*g/day	Parenteral PDE,*μ*g/day	Inhalation PDE,*μ*g/day
Cd	1	5	2	3
Pb	1	5	5	5
As	1	15	15	2
Hg	1	30	3	1
Co	2A	50	5	3
V	2A	100	10	1
Ni	2A	200	20	5
Tl	2B	8	8	8
Au	2B	100	100	1
Pd	2B	100	10	1
Ir	2B	100	10	1
Os	2B	100	10	1
Rh	2B	100	10	1
Ru	2B	100	10	1
Se	2B	150	80	130
Ag	2B	150	10	7
Pt	2B	100	10	1
Li	3	550	250	25
Sb	3	1200	90	20
Ba	3	1400	700	300
Mo	3	3000	1500	10
Cu	3	3000	300	30
Sn	3	6000	600	60
Cr	3	11000	1100	3

**Table 2:** Accuracy of 10 elements in parecoxib sodium.

Analyte	Added (*μ*g/L)	Found (*μ*g/L)	Recovery (%)
Cd	0.2 (50%)	0.183, 0.190, 0.192	91.0, 94.5, 95.5
	0.4 (100%)	0.362, 0.363, 0.364	90.2, 90.5, 90.7
	0.6 (150%)	0.568, 0.573, 0.560	94.5, 95.3, 93.2
	Average	—	92.8

Pb	0.5 (50%)	0.515, 0.519, 0.528	103.0, 103.8, 105.6
	1 (100%)	1.053, 1.010, 1.021	105.3, 101.0, 102.1
	1.5 (150%)	1.576, 1.596, 1.553	105.1, 106.4, 103.5
	Average	—	104.0%

As	1.5 (50%)	1.804, 1.799, 1.740	120.1, 119.7, 115.8
	3 (100%)	3.348, 3.453, 3.410	111.5, 115.0, 113.6
	4.5 (150%)	5.238, 5.168, 5.122	116.3, 114.8, 113.8
	Average	—	115.6%

Hg	0.3 (50%)	0.295, 0.298, 0.302	98.3, 99.3, 100.7
	0.6 (100%)	0.636, 0.628, 0.649	106.0, 104.7, 108.2
	0.9 (150%)	1.005, 1.009, 0.990	111.7, 112.1, 110.0
	Average	—	105.7%

Co	0.5 (50%)	0.545, 0.552, 0.510	108.6, 110.0, 101.6
	1 (100%)	1.003, 1.034, 1.034	100.1, 103.2, 103.2
	1.5 (150%)	1.591, 1.571, 1.527	105.9, 104.6, 101.7
	Average	—	104.3%

V	1 (50%)	1.167, 1.173, 1.099	116.0, 116.6, 109.2
	2 (100%)	2.139, 2.207, 2.183	106.6, 110.0, 108.8
	3 (150%)	3.364, 3.312, 3.312	111.9, 110.2, 110.2
	Average	—	111.1%

Ni	2 (50%)	2.366, 2.344, 2.749	110.5, 109.6, 129.9
	4 (100%)	4.099, 4.495, 4.192	98.8, 108.8, 101.1
	6 (150%)	6.411, 6.289, 6.143	104.3, 102.3, 100.1
	Average	—	107.3%

Li	25 (50%)	27.990, 28.433, 26.886	111.9, 113.7, 107.5
	50 (100%)	53.937, 54.078, 54.799	107.8, 108.1, 109.6
	75 (150%)	83.850, 82.878, 82.051	111.8, 110.5, 109.4
	Average	—	110.0%

Sb	9 (50%)	8.362, 8.339, 8.962	92.9, 92.7, 99.6
	18 (100%)	16.430, 16.794, 16.614	91.3, 93.3, 92.3
	27 (150%)	26.007, 25.247, 25.703	96.3, 93.5, 95.2
	Average	—	94.1%

Cu	30 (50%)	32.150, 32.031, 30.808	107.1, 106.7, 102.7
	60 (100%)	59.092, 61.518, 60.352	98.5, 102.5, 100.6
	90 (150%)	94.354, 92.470, 91.905	104.8, 102.7, 102.1
	Average	—	103.1%

**Table 3:** Precision of 10 elements in parecoxib sodium.

Matrix	*Recovery (%)*									
	Cd	Pb	As	Hg	Co	V	Ni	Li	Sb	Cu
Interday	92.0	102.3	116.8	110.0	110.2	118.1	107.3	113.6	93.3	104.3
	92.8	103.9	115.7	111.3	106.7	114.0	103.9	110.5	93.5	101.5
	96.7	103.7	115.7	110.0	110.9	118.2	109.9	111.0	93.7	104.9
	95.5	101.3	116.2	109.3	112.1	119.6	108.2	110.6	92.0	106.7
	91.2	103.7	118.4	110.2	109.6	119.0	106.8	112.4	92.5	105.5
	95.0	100.9	114.5	109.2	108.8	117.2	106.3	111.3	92.0	104.1

Intraday	93.5	100.9	116.9	106.2	110.4	116.4	108.9	110.4	94.7	106.4
	90.8	103.3	113.8	105.0	110.9	116.1	105.6	111.2	92.2	103.5
	94.3	103.4	116.1	109.0	112.2	117.0	111.7	110.1	94.6	107.2
	92.5	100.1	117.1	105.0	111.2	118.3	108.1	109.7	93.9	106.8
	94.8	106.3	119.4	110.7	112.6	121.2	111.1	112.6	94.5	108.9
	93.3	104.3	119.8	109.0	113.0	120.1	109.8	113.1	94.6	108.9

RSD (%)	2.0	1.8	1.6	2.0	1.7	1.7	2.2	1.2	1.2	2.1

## Data Availability

The data used to support the findings of this study are included within the article.

## References

[1] Barton S. F., Langeland F. F., Snabes M. C. (2002). Efficacy and safety of intravenous parecoxib sodium in relieving acute postoperative pain following gynecologic laparotomy surgery. *Anesthesiology*.

[2] Malan T., Marsh G., Hakki S., Grossman E., Traylor L., Hubbard R. (2003). Parecoxib sodium, a parenteral cyclooxygenase 2 selective inhibitor, improves morphine analgesia and is opioid-sparing following total hip arthroplasty. *Anesthesiology*.

[3] Cheer S. M., Goa K. L. (2001). Parecoxib (parecoxib sodium). *Drugs*.

[4] Smith R. J., Webb M. L. (2014). Analysis of drug impurities. Tailieu vn. https://www.google.com/search?q=Analysis+of+Drug+Impurities+2014&rlz=1C1GCEJ_enIN1016IN1016&ei=yT_7YuaQA4LCz7sP57OVmAU&ved=0ahUKEwimmaaQ5Mr5AhUC4XMBHedZBVMQ4dUDCA4&uact=5&oq=Analysis+of+Drug+Impurities+2014&gs_lcp=Cgdnd3Mtd2l6EAMyBQghEKABOgcIABBHELADOgYIA.

[5] Guideline I. (2004). Impurities in New drug substances. *Q3a*.

[6] Guideline (2009). Impurities in new drug products. https://www.ema.europa.eu/en/ich-q3b-r2-impurities-new-drug-products.

[7] Yong-Qi S. U., Pei-Si L. I., Ren L. L., Guo X. D., Wu Y. L. (2010). Determination of chromium in milk powder by ICP-MS combined with microwave digestion. *Modern Food Science and Technology*.

[8] Millour S., Noël L., Kadar A., Chekri R., Vastel C., Guerin T. (2011). Simultaneous analysis of 21 elements in foodstuffs by ICP-MS after closed-vessel microwave digestion: method validation. *Journal of Food Composition and Analysis*.

[9] Pereira J. S., Moraes D. P., Antes F. G. (2010). Determination of metals and metalloids in light and heavy crude oil by ICP-MS after digestion by microwave-induced combustion. *Microchemical Journal*.

[10] Gonzalez M. H., Silva C. S. D., Amaral C. D. B. (2016). Determination of elemental impurities in acyclovir ointment and raw materials using microwave acid digestion (MW-AD) and ICP-MS. *Journal of the Brazilian Chemical Society*.

[11] Gredilla A., de Vallejuelo S. F. O., Arana G. (2022). A rapid routine methodology based on chemometrics to evaluate the toxicity of commercial infant milks due to hazardous elements. *Food Analytical Methods*.

[12] Teasdale A., Elder D., Nims R. W. (2017). *ICH Q3D Elemental Impurities*.

[13] Cui X. S., Chen Z. Y., Zeng H. X., Pan W. S. (2017). Development and validation of the production process of parecoxib sodium freeze-dried preparation based on quality by design. *Chinese Pharmaceutical Journal*.

[14] Elder D., Guidelines I. (2013). Ich q6a-specifications: test procedures and acceptance criteria. https://www.gmp-compliance.org/files/guidemgr/3-1-16.pdf.

